# VEMERS 2.0: Upgrading of an Emergency Use Ventilator from a Single Mandatory Volume Control Mode of Ventilation (VEMERS 1.0) to 8 Modes of Ventilation

**DOI:** 10.1155/2022/6965083

**Published:** 2022-06-06

**Authors:** Luciano E. Chiang, Felipe A. Castro, Tomás F. Sánchez

**Affiliations:** Department of Mechanical Engineering, Pontifical Catholic University of Chile, Vicuna Mackenna Avenue 4860, Comuna Macul, Region Metropolitana, Chile CP 7820436

## Abstract

The upgrading of an emergency use ventilator from a single mandatory volume control mode of ventilation (VEMERS 1.0) to 8 modes of ventilation (VEMERS 2.0) is described. The original VEMERS 1.0 was developed in the midst of the COVID-19 crisis in Chile (April to August 2020) following special but nonetheless strict guidelines specified by local medical associations and national health and scientific ministries. The upgrade to 8 modes of ventilation in VEMERS 2.0 was made possible with minor but transcendental changes to the original architecture. The main contribution of this research is that starting from a functional block diagram of an ICU mechanical ventilator and carrying a systematic analysis, the main function blocks are implemented in such a way that combinations of standard off-the-shelf pneumatic and electronic components can be used. This approach has both economical and technical advantages. No special parts need to be fabricated at all, and because of a wider variety of options, the use of extensively field-proven off-the-shelf commercial components assures better availability and lower costs when compared to that of conventional ICU mechanical ventilators, without sacrificing reliability. Given the promising results obtained with VEMERS 2.0 in the subsequent national certification process, the production of 40 VEMERS 2.0 units was sponsored by the Ministry of Science and the Ministry of Economy. Twenty units have been distributed among hospitals along the country. The purpose of VEMERS 2.0, as a low-cost but very reliable option, is to increase the number of mechanical ventilators available (3,000 for a population of 18,000,000) in the country to eventually reach a ratio similar to that of more developed countries. VEMERS is an open-source project for others to use the knowledge gained.

## 1. Introduction

COVID-19 was designated as a pandemic in 2020 by the WHO. The high number of active cases, more than 209.000.000 and more than 4.400.000 deaths in the world at the time this article was written [1], has overstressed health systems all over the world. From these, in Chile, more than 1.630.000 cases with 36,605 deaths have been reported [2]. A vital resource for treating patients with respiratory problems caused by COVID-19 is mechanical ventilators.

In Chile, at the beginning of the pandemic, there were 1.229 mechanical ventilators [2]. Moreover, Chile reached a peak of almost 90.000 active cases [2] in June 2020. The evolution of UIC beds and occupancy are shown in Figure 1 [2]. At the maximum peak, there were 3,000 mechanical ventilators in use (“Pctes. UCI COVID 19 en VMI”), and the capacity of the health system was close to 100% for a long period of time (April-June, 2021), meaning that in practice there must have been regional shortages and many patients had to be transported to accommodate for site availability.

In fact, there was a localization problem since the geographic distribution of mechanical ventilators and trained personnel, generated shortages in regional hospitals as the active cases in geographic distribution evolved.

In March 2020, at the beginning of the COVID-19 pandemic in Chile, many ideas had been made available publicly already in the world to face the shortage of mechanical ventilators [3, 4]. Many open-source solutions were proposed, some based on the mechanization of bag-mask manual ventilators [5–7], and others followed an electropneumatic principle [8–10]. Existing solutions such as E-vent [5], OxVent [6], and OxyGEN [7] were rapidly adopted by local developers in Chile, and many propositions were submitted to local authorities. Very few are known to have achieved any clinical validation both in Chile and in the world.

The entity in Chile that certifies health products, ISP (Public Health Institute), was not prepared to certify sophisticated medical equipment such as emergency mechanical ventilators. Contacts between government ministries, scientific societies, and professional and industry associations gave rise to the Multidisciplinary Council for Facilitation and Management of the COVID-19 Crisis (CMFCC) to fill the void. Its members were all appointed voluntarily and acted pro-bono. The CMFCC asked three medical societies: Chilean Society of Intensive Medicine (Sociedad Chilena de Medicina Intensiva (SOCHIMI)), Chilean Society of Urgency Medicine (Sociedad Chilena de Medicina de Urgencia (SOCHIMU)), and the Chilean Society of Anesthesiology (Sociedad de Anestesiología de Chile (SACH)), to issue a protocol to validate emergency mechanical ventilators, which could later be produced in large scale. The final version of the protocol was published on June 3, 2020 [11], but preliminary versions had begun circulating much earlier. At the same time, the CMFCC issued a call for proposals and preselected 5 initiatives to guide in the process of validation. Initiatives that were not selected or of later appearance were allowed to follow the process but subject to the availability of the authorized validation entities. VEMERS UC came in late but decided to follow the process because validation in an open process would give the ventilator much more credibility. In the end, it was the right decision because the government announced a few weeks later that it would only consider funding proposals that complied with the validation protocols issued by the CMFCC. In addition, MHRA (UK) [12], AAMI (USA) [13], and also ISO 80601-2-12 [14] design guidelines have also been taken into account. For the most part, it can be said that protocols [11–13] are quite similar to each other since they have been specifically tailored for emergency mechanical ventilators to be used during the COVID-19 pandemic. In fact, VEMERS 1.0 [15] after completing the CMFCC validation process has received 2 grants, one private and another from the government to produce 40 units in total.

In the following sections, the technical aspects of VEMERS 2.0 upgrading will be described in detail.  Figure 2 shows the two versions developed so far.  Table 1 shows the general ranges of operation of VEMERS 2.0. This article is useful because it shows how an EUV can be upgraded and left available for general postpandemic use, especially in low-resource communities.

The COVID-19 pandemic has made patent the shortcomings of ICU services in the world health system, particularly in low resource settings. It has become clear that there is only a shortage of mechanical ventilators but there is also a shortage of respiratory therapists that can operate correctly and safely these systems which can be very complex. There are situations that generate confusion and hence risk situations even to the most experienced RTs. According to recent studies [16–18], the main directions in the future development of mechanical ventilators are as follows:

- Mechanical ventilators should maintain their functionality and capabilities or even increase them, but personnel with less experience and training should be able to operate them safely as well. This requires adding intelligent and real-time processing of the ventilator output signals to help guide the operator through situations that arise than can be confusing for the nonexpert. This would require, for example, automation of the ventilator settings, something that in the present state of the art is done manually, hence, including intelligent decision-making systems and big data processing capabilities.
- The user interface should be easy to understand and configure. The interpretations of warnings and alarms when occurring simultaneously should be processed quickly so that it is easier to stabilize the patient, reducing risks. The ventilator must take automatic corrective actions in specific situations of high risk, especially if there is a mechanical ventilator part failure causing this situation. Hence, reliability is an issue that must continuously improve.
- The ventilators should be teleoperated at a distance so that the RT does not have to come into close contact with the patient unless it is necessary. This would also allow the RT to handle more patients at one time, because it would take less time to check periodically a patient, saving time in such pedestrian chores as getting dressed, for example.

## 2. Methods

### 2.1. Choked Inhalation AirFlow

Both VEMERS 1.0 and VEMERS 2.0 rely on generating a choked flow [19] from the air mixture source to the ventilator inspiratory branch. A choked flow allows regulating the inhalation flow by controlling the opening of a flow control valve only, thus simplifying the construction of the ventilator.

To better understand this, let us consider the system in Figure 3. Reservoir 0 is in stagnant conditions *p*_0_,  *T*_0_,  *ρ*_0_. The flow through *A*_1_ will depend on the value of *p*_2_ (see Nomenclature table). Index 2 refers to the patient's lungs. Hence, as long as

(1) $$\begin{array}{c} p_{2}\leq p^{*}=p_{0}{\left(\frac{2}{k+1}\right)}^{k/k-1}\;, \end{array}$$

then the pressure *p*_1_ will be always

(2) $$\begin{array}{c} p_{1}=p^{*}=p_{0}{\left(\frac{2}{k+1}\right)}^{k/k-1}. \end{array}$$

If this is the case, then the flow through *A*_1_ that enters reservoir 2 is fixed regardless of the value of *p*_2_and is given by the following expression:

(3) $$\begin{array}{c} {\dot{Q}}_{1}=A_{1}\sqrt{2\frac{\;c_{p}}{R}p_{0}\rho_{0}{\left(\frac{k-1}{k+1}\right)}^{k-1/k}}. \end{array}$$

From the above equation, it is clear that if the stagnant conditions in reservoir 0 remain constant, then the flow entering reservoir 2 (patient lungs) depends exclusively on the magnitude of the section area *A*_1_. If the section area *A*_1_ is set using a proportional flow control valve as in VEMERS 2.0 or a manual flow control valve as in VEMERS 1.0, then the actual flow going into reservoir 2 can be also accurately fixed. This is the principle used in both VEMERS versions in the inspiratory phase of the respiratory cycle. The inspiratory phase is achieved with a choked airflow since the pressure in reservoir 0 is kept at 2 bar and at ambient temperature, while the pressure in reservoir 2 (i.e., the patient) never rises above 60 cm H20 (thus *p*_2_ is always much less than *p*^*∗*^).

### 2.2. Control of Exhalation Flow

The expiratory flow is governed by the same compressible gas flow equations. The patient's lung is in varying conditions *p*_2_,  *T*_2_,  *ρ*_2_ as shown in Figure 4. It is connected to the ambient air at atmospheric pressure *p*_*a*_ through the expiratory branch which has an aperture section area *A*_3_. The magnitude of patient lung pressure *p*_2_ is such that the corresponding critical pressure *p*^*∗*^ is always lower than *p*_*a*_. Hence, the pressure at section *A*_3_ (the expiratory valve aperture) will be *p*_*a*_ rather than *p*^*∗*^.

The flow through *A*_3_ is thus governed by the following equation:

(4) $$\begin{array}{c} {\dot{Q}}_{3}=A_{3}\sqrt{\left(p_{2}-p_{a}\right)\rho_{2}}. \end{array}$$

A PID control loop of the section area *A*_3_ aperture allows quickly driving *p*_2_ to the desired peep value and keeping its variation within acceptable limits.

### 2.3. Electropneumatic Upgrade

The main upgrade done to the electropneumatic circuit in VEMERS 1.0 (shown in Figure 5) has been the replacement of both the inspiratory and expiratory valves [15]. These two valves in the emergency mechanical ventilator version VEMERS 1.0 were directional 2 × 2 on-off valves. In the upgraded version VEMERS 2.0, they have been replaced by proportional 2 × 2 valves. VEMERS 1.0, as a basic EUV, has only one mode of ventilation, namely, volume control mode. The implementation of the volume control mode of ventilation (VC) alone is satisfied using only on-off directional valves. The inspiratory phase in the case of VEMERS 1.0 is implemented in combination with a manual choke valve since this allows setting a fixed magnitude inspiratory flow, which is characteristic of this mode of ventilation.

However, to implement pressure control mode, it is necessary to use a proportional valve in order to continuously adjust the airflow to reach and maintain the desired pressure level, which is characteristic of the pressure control mode and its variants. This has been done in VEMERS 2.0.

On the other hand, the expiratory phase of the volume control mode cycle in VEMERS 1.0 [15] was implemented by using four 2 × 2 directional valves, which were activated in sequence in order to quickly reach and maintain the desired peep pressure values. In this case, the four valves are open at the beginning of the expiratory phase, and each one is closed sequentially according to the pressure level. In this manner, the pressure level quickly falls at the beginning of the expiration, and when the pressure is close to the desired peep value, they are closed in sequence to reduce the expiratory flow to the minimum necessary value.

In VEMERS 2.0, these four valves are replaced by a single proportional valve (SPV2), which allows controlling the expiratory flow so that the pressure quickly falls at the beginning of the expiration and later closes just enough to maintain the peep pressure at the end of the cycle.

The respirator has two intakes, one for air and one for oxygen supply. In a standard hospital ICU, both gases are available at 50 psi in wall faucets. In the schematics in Figure 6, pressure sensors S5 and S6 detect the correct supply of gases. Each gas line then enters a pressure regulator (PRV1 and PRV2) that set pressure outputs to a value of two bar so the oxygen-air mix (FiO2) can be set properly.

#### 2.3.1. Blending Stage

Each gas line enters next to a manual flow control valve arrangement (FCV2 and FCV3). Both valves are connected head to head, allowing the setting of the FiO2 by a common knob. Turning this knob will open one valve and at the same time close the other. This allows controlling in a very simple and reliable way the resulting FiO2 because the RT can check its value on the computer screen and adjust the knob by hand. The air and O2 are then mixed between 21% (standard air) and 100% of oxygen as set by the RT before passing through electropneumatic proportional valve SPV1. The scheme implemented in VEMERS provides a low-cost, reliable, and immediately available solution for gas mixing.

#### 2.3.2. Inspiratory Stage

The gas mixture passes through a 2 × 2 proportional solenoid valve (SPV1) which is opened in the inspiratory phase and closed in the expiratory phase commanded by a PWM controller signal. A PID control loop allows reaching either a set volume or a set pressure depending on the mode of ventilation. There is a choking effect which is a key feature because it allows the inspiratory gas mixture flow rate to be independent of the discharge pressure downstream of SPV1 and only dependent on the aperture level commanded by the PWM control circuit. In volume control mode, the inhalation gas flow rate remains constant and is adjusted so that the desired tidal volume is reached. In pressure control mode, the aperture of SPV1 is continuously set such that the pressure in the inhalation branch is maintained at the desired level.

Differential pressure sensor S1 allows monitoring the instantaneous pressure in the breathing circuit from −100 to 100 MPa. This sensor is also used to detect patient triggering. Sensor S2 is a galvanic oxygen sensor that allows measuring FiO2. This type of galvanic sensor is the same commonly used in full-fledged high-end ventilators. They have a low-time response. Hence, in VEMERS UC, the RT must wait a few seconds until the oxygen sensor signal stabilizes to verify on the computer screen that the desired value has been reached.

Unidirectional flow sensor S3 measures the inspiratory flow in a range from 0 to 200 lpm, as it leaves through the inspiratory port where the inspiratory tubing leading to the endotracheal tubing is connected.

#### 2.3.3. Exhalation Stage

In VEMERS 2.0, the exhalation stage is controlled by a solenoid 2 × 2 proportional valve (SPV2). The controller reads pressure sensor S1 and activates the SPV2 valve according to a PID control scheme that sends a PWM signal to SPV2. The pressure must quickly drop to the desired peep value and later maintained stability.

A HEPA filter and water trap are commonly installed in this line in between the ventilator and the endotracheal tube.

### 2.4. Software Upgrade

VEMERS 1.0 as an emergency mechanical ventilator was developed with only one mode of ventilation (mandatory volume control). VEMERS 2.0 has been upgraded to 8 modes of ventilation with the architecture shown in Figure 6 and additional ad hoc user interface and control software. As the COVID-19 treatment evolves in patients, different modes of ventilation may be more convenient, as well as for respiratory diseases other than COVID-19 [20]. The 8 modes of ventilation are listed in Table 2.

#### 2.4.1. Ventilation Modes

In this section, a brief description of the ventilation modes available in VEMERS is given. We do not intend to give a complete and extended discussion because of limitations of space and the complexity of the subject, but the reader can be referred to [20] for a detailed in-depth discussion of these modes which are well known in the critical care medical community.

*Mode 1. Volume Control Mode*. This is a mandatory invasive mode of ventilation. The respirator essentially delivers a constant volume of air (the tidal volume) to the patient at a fixed frequency in each cycle according to the preset values. For this mode of ventilation to work properly, the inspiratory flow must be controlled to a high degree of accuracy so that at the end of the cycle the desired air volume is precisely delivered. The patient is not allowed to initiate a respiratory cycle on its own. In the expiratory phase, the output flow is controlled to maintain the airway pressure at the desired PEEP level, which is a safe level to avoid patient alveoli collapse.

In this mode of ventilation, the following parameters must be set by the RT.

- Tidal Volume (ml)
- PEEP (cmH20) (positive end-expiratory pressure, the minimum pressure allowed in the respiratory system)
- Respiratory Frequency (bpm)
- I : E ratio (the ratio between inspiratory time and expiratory time in the cycle)
- FiO2 (%) percentage of additional oxygen in the air mixture delivered to the patient
- Plateau time/inspiratory pause. The interval of time in which the flow is paused during the inspiration phase (s)
- PIP maximum pressure allowed in the respiratory cycle

Figure 7 shows the characteristic shapes of patient curves in volume control mode.

*Mode 2. Assisted Volume Control*. This mode of ventilation is similar to the above except that if the patient attempts to initiate a respiratory cycle on its own (asynchronously) during the exhalation phase, the respirator will immediately deliver a new cycle provided that the negative pressure level generated by the patient has met a minimum threshold. The triggering pressure is set by the RT.

*Mode 3. Pressure Control Mode of Ventilation*. In Pressure Mode of ventilation, the pressure in the respiratory system is maintained at a desired fixed level during the inspiratory phase. As a result, the pressure curves should look like a square train pulse. In the exhalation phase, the ventilator must reach and maintain the pressure at the desired PEEP value. In this mode, the ventilator controls the inspiratory flow starting with a high flow value and then reducing it as pressure rises and reaches the set value. The variables to set in this mode of ventilation are the following:

- P insp [cmH2O]
- PEEP [cmH20]
- Frequency (bpm)
- IE ratio
- Fraction of inspiratory oxygen FiO2 [%]

Figure 8 shows characteristic curves obtained in pressure control mode.

*Mode 4. Assisted Pressure Control*. This mode of ventilation is similar to the above (see 2.4.1.3) except that if the patient attempts to initiate a respiratory cycle on its own (asynchronously) during the exhalation phase, the respirator will immediately deliver a new cycle provided that the pressure level generated by the patient has met a minimum threshold. The triggering pressure is set by the RT.

*Mode 5. Pressure Support Mode of Ventilation*. This mode of ventilation is used to facilitate the patient's transition to autonomous breathing prior to disconnection from the ventilator. In this mode, the respirator will wait until the patient attempts a breathing cycle. If the waiting time (T apnea) is surpassed, then the ventilator switches back automatically to mandatory volume control. However, if there is a patient effort strong enough, inspiratory flow is allowed, maintaining a fixed support pressure until the flow reduces to a fraction of the initial maximum, and at this moment, the ventilator switches to the expiratory phase. Hence, in this mode, the ventilator lets the patient set the respiratory pace, allowing a gradual process of autonomous breathing before disconnection. The amount of air that is delivered is proportional to the patient's effort.

- IE ratio
- PEEP [cmH20]
- FiO2 [%]
- ∆ support pressure [cmH20] above PEEP level
- Trigger pressure [cmH20] below PEEP level)
- Frequency in safety volume control mode [bpm]
- Tidal volume in safety volume control mode [ml]
- T apnea [s] (waiting time before switching to safety volume control mode).

Figure 9 shows typical patient curves in pressure support mode.

*Mode 6. CPAP (Continuous Positive Airway Pressure)*. Modes 6 to 8 are nonintubated modes of ventilation that have proven to be useful for standby patients before intubation. In Mode 6, the patient receives a constant positive airway pressure through a breathing mask. The value of the pressure is set by the RT and it is always constant regardless if the patient is in the inspiratory or expiratory phase. The parameters that need to be set in this mode are as follows:

- CPAP [cmH20]
- FiO2 [%]

Figure 10 shows typical curves for this mode.

*Mode 7. BiPAP (BiLevel Positive Airway Pressure)*. This ventilation mode consists in providing the patient with two levels of pressure during a respiratory cycle. In the inspiratory phase, the pressure level is higher while in the expiratory phase the pressure is set to a minimum value to facilitate expiration but avoid the risk of the collapse of the patient's alveoli.

The operating parameters that must be set in this mode are the following:

- High level Bipap pressure [cmH2O]
- Low level Bipap pressure [cmH20]
- Respiratory Frequency (cpm)
- IE ratio Razón I : E (1:N)
- FiO2 (%)

Figure 11 shows typical patient curves for this mode.

*Mode 8. High-Flow Nasal Cannula Oxygenation*. In this mode of ventilation, a constant high flow of pure oxygen or air oxygen mixture is delivered to the patient by way of a cannula entering the nose of the patient. The parameters that must be set in this mode of ventilation are as follows:

- Flow [L/min]
- FiO2 [%]

Figure 12 shows patient curves in this mode of ventilation.

### 2.5. User Interface

VEMERS 2.0 has an internal microcontroller to synchronize the respiration cycle. In addition, it includes a touch screen computer that communicates with the internal microcontroller so the RT can set the cycle parameters. Hence, in the case of VEMERS 2.0, both the internal microcontroller and touchscreen interface computer software are much more complex than in VEMERS 1.0. The internal microcontroller software is written in C++. The user interface software in the touchscreen computer is written in C#.

User interface screens are shown in Figures 13–15. The interface has common features for all modes of ventilation as well as specific individual ones. The text in all user interfaces is in the Spanish language because the RT in Chile prefers to set the ventilator in the native language. At the left of the user screen, all modes of ventilation show 3 real-time graphs from top to bottom: pressure, flow, and volume. The mode of ventilation is selected using the proper radio buttons in the boxes with pink and brown backgrounds. Each mode of ventilation has individual input parameters to be set, and output parameters that can be read. The input parameters set by the RT are in the green background boxes. In these, the interior textboxes with the white background are the input parameters entered by the RT, and the inner textboxes in grey give the actual instantaneous values. The cycle output parameters are in the boxes with the cyan background. There is a message box (“Mensajes”) in the middle of the screen with a white background that generates error messages when anomalies are detected. There is also a dropdown menu of options to set general operational alarm limits (“Menu Opciones”).

## 3. Results and Discussion

### 3.1. Design Issues

The electropneumatic proportional valves are arguably the most important parts of VEMERS 2.0. At the height of the pandemic, these valves were extremely difficult to find. The cost is also 10–100 times that of the combination of a directional valve plus a manual flow control valve used in VEMERS 1.0. The cost of the proportional valves used in VEMERS 2.0 is in the order of USD 250 each. Nevertheless, even though the cost of parts and materials to assemble VEMERS 2.0 increases from USD 1,750 [15] in VEMERS 1.0 to USD 2,000, this is a fraction of the price of a conventional high-end mechanical ventilator commercially available.

The selection of the electropneumatic valve is key to the correct functionality and reliability of the mechanical ventilator as a whole. Shown in Figure 16 is the valve flow versus PWM behavior of two proportional valves. The wider range of valve SMC 2121-3 allows much better and more reliable control of the operation of the ventilator. A narrower range gives rise to a jumpy response; hence, the respiratory parameters oscillate more.

### 3.2. Technical Certification

Both VEMERS 1.0 and VEMERS 2.0 have been thoroughly tested, so they can be used safely and with confidence.  Table 3 gives validations that have been performed on both VEMERS 1.0 and VEMERS 2.0.

A brief description of tests.

#### 3.2.1. Technical Validation Tests 1 and 4

Starting tests were the technical validation tests. The main objectives of these tests were as follows:

- Accuracy verification in individual incremental parameter setting in volume control mode of ventilation, that is to say, verification of parameter accuracy in individual incremental setting of tidal volume, PEEP, and frequency.
- Accuracy verification in the combinatorial setting of working parameters in volume control mode of ventilation
- Documentation Revision
- Equipment Labeling Revision
- Alarm Verification
- Electric safety verification

The methodology for technical validation at the certification bureau (Certemed) consisted of connecting the ventilator prototype to an Acculung II Fluke test lung with a Fluke VT650 gas analyzer in between. Single parameters were incremented individually according to a predefined sequence, and the accuracy of VEMERS UC readings was assessed as explained above in (a). Next, different combinations of working parameters were tested according to a predefined sequence, and the accuracy of VEMERS UC readings was compared. In all, more than 450 tests and verifications are required in this technical evaluation.

The technical evaluation protocol includes a list of alarms that had to be implemented and activated in a correct and timely manner. Using a Umik-1 microphone, the sound level of the alarms is measured, which must be at least 6 dB above ambient noise.

To check electrical safety, a Fluke ESA 620 was used. This instrument is certified to measure ground protection impedance, ground current leakage, and envelope leakage current.

#### 3.2.2. Test 2: Usability

A usability evaluation was required. The VEMERS UC development team was asked to make an online presentation to a panel of experts consisting of written documentation and videos explaining the principle of operation of VEMERS UC and the user interface. User-friendliness, readability of the screen, respiratory parameter settings, quality of knobs and switches, among others were of paramount importance to obtain approval in this test. The assembly process of VEMERS UC was also discussed to assess production time and cost.

#### 3.2.3. Preclinic Tests

Preclinic tests were carried out at the Center for Medical Research of the Pontifical Catholic University of Chile. The objectives of these tests were as follows:

- Verify the functionality and capability of modifying ventilation parameters
- Verify compliance of programmed and resulting ventilation parameters (tidal volume, PEEP, I/*E* ratio, inspiratory pressure)
- Evaluate correct functioning of alarms
- Verify that the ventilator prototype maintains an effective gas exchange in a healthy model as well as in a model with pulmonary injury
- Verify that the ventilator prototype is capable of maintaining a protective ventilation (volume 6 ml/kg, plateau pressure <30 cmH2O, DP < 15) in a model with pulmonary injury

The methodology in these tests consisted of the use of a porcine animal model, subject to 2 consecutive experimental sequences: (i) tests on the healthy model and (ii) tests on the model with induced pulmonary injury.

VEMERS UC preclinic tests proved compliance with all the important aspects in providing ventilation and maintaining a gaseous exchange similar to a conventional mechanical ventilator under normal as well as in the case of moderately altered pulmonary function.

#### 3.2.4. Clinical Tests with COVID-19 Patients

Clinical tests were performed on 5 COVID-19 patients at the Clinical Hospital of the Catholic University of Chile. The objectives of these tests were as follows:

- Evaluate the safety and effectiveness of VEMERS UC for use in patients with acute pulmonary pathology
- Evaluate the capacity of VEMERS UC to maintain the gaseous exchange and cardiovascular safety in critically ill patients with pulmonary pathology for stretches of 8 hours

The methodology in these tests was to find patients with a relation PaO2/FiO2 (PaFi) between 100 and 250, having vasopressor support with Norepinephrine <0.2 *μ*/kg*∗*min, and with medical indications of deep sedation and muscle blockage. The test consisted of measurements of oxygenation and cardiovascular parameters during operation. For each patient, the first 2-hour measurements were every 15 minutes and after that every 1 hour. The working parameter settings in VEMERS UC were the same as the patient had with the conventional ventilator previously connected (Table 4). Patient General Data in VEMERS UC Clinical tests contain general patient data in the tests.

The clinical tests on VEMERS UC showed that it is capable of safely maintaining oxygenation and PaCO2 exchange. It can provide protective ventilation and gas exchange similar to a traditional mechanical ventilator under conditions of impaired lung function. Since this was the last test specified in the CMFCC protocol [18], after completion, this council issued a final report of overall approval.

#### 3.2.5. Advanced Technical Evaluation

There are specific tests for advanced volume control mode of ventilation, as well as pressure control mode of ventilation. In the pressure control mode of ventilation, the most complex set of tests is to verify trigger levels for Pressure Support Systems. Otherwise, the tests are quite similar as described in Section 3.2.1.

### 3.3. Reliability

VEMERS 1.0 was tested clinically with five COVID-19 intubated patients for 8 hours each [24]. To further verify the reliability, one VEMERS 2.0 unit was set apart for long-term testing. That unit has been running nonstop in different ventilation modes starting on April 23, 2021, using a test lung. At the moment of writing this article, it had been running for 121 straight days without any failure. Patients usually stay connected to a mechanical ventilator for not longer than one month. Hence, this demonstrates the robustness of the VEMERS design.

It is surprising from an engineering point of view that extensive reliability tests are not required to certify a mechanical ventilator. This aspect seems to be left to the responsibility of the manufacturer. This is probably why brand recognition in the mechanical ventilator market is so important. The special set of standards for emergency use ventilators recommended by [12] is the only standard that specifically requires demonstrating the continuous operation of 14 days. The most cited document relative to certification of conventional high-end ventilators published by the WHO [14] does not contain any requirements in terms of reliability. In Chile, throughout the pandemic, a number of units of lesser-known brands failed prematurely, which is why the authors think that reliability should be considered in more depth and detail for certification purposes in the future.

### 3.4. Unit Distribution

At the time of writing this article, 20 VEMERS 2.0 units have been distributed in the Chilean national health system among 9 hospitals as shown in Table 5.

Usage of VEMERS 2.0 has been mainly as backup units and mostly in patients in noninvasive ventilation modes (CPAP, BiPAP, and High Oxygen Flow Therapy) in emergency rooms of hospitals. Given the nature of this medical equipment and the evolution of the COVID-19 pandemic, clinical testing of VEMERS 2.0 has required much more time than expected. More technical and user updated information can be found on http://www.vemers.cl, or on the VEMERS YouTube channel.

## 4. Conclusions

An emergency use ventilator VEMERS 1.0 was previously developed to comply with the Chilean requirements specified by CMFCC, an ad hoc task force formed by several medical associations, government offices, and industry leaders in Chile. VEMERS 1.0 also complies with MHRA [12] and AAMI [13] guidelines, according to internal tests performed. As an emergency use ventilator, VEMERS 1.0 is only required to work in a mandatory volume control mode of ventilation. In this article, VEMERS 2.0 is described, which was expanded to eight different ventilation modes by replacing previous directional electropneumatic valves with proportional valves. This allows not only direct flow control but also pressure control, thus making additional modes of ventilation possible. Proportional valves are more expensive and more difficult to find than directional valves, but they allow not only to expand the capabilities of the original VEMERS 1.0 but also to automate the setting of the respiratory cycle possible, since manual flow control valves are then not needed. The expansion of capabilities in VEMERS 2.0 has been certified by a Chilean authorized certification bureau (Certemed).

Twenty VEMERS 2.0 units have been distributed within the Chilean national health system. These units have remained as backup and are used occasionally now that the COVID-19 pandemic has receded, and that the Chilean health system has enough conventional mechanical ventilators to satisfy demand.

VEMERS 2.0 can be produced buying all its components in the general industrial pneumatic market, and there is really no component that needs to be specially fabricated. The production is mainly an assembly process that takes around 1 day. The approximate cost of the components in Chile is USD 2,000, which is much less than that of high-end mechanical ventilators today in the market. Considering the fact that the general resources in Chile as well as in many other countries cause less than ideal availability of medical equipment, the knowledge and experience gained in the VEMERS project can be helpful to counter this situation.

However, it is important to keep in mind that being VEMERS, a life-supporting device, there are high risks in using consumer/industrial grade electronics and components, although they may be appropriate as an absolute last resort in the absence of alternative medical grade options during the current pandemic. For this reason, additionally, VEMERS parts and as a whole are being thoroughly and continuously tested to anticipate situations of failure. Until now, VEMERS architecture and components have been reliable. In spite of having a smaller set of modes of ventilation than some conventional high-end mechanical ventilators, its demonstrated reliability and functionality are a good solution for the majority of situations that a patient with respiratory problems such as COVID-19 will face.

Thus, the main contribution of this research that can be stated is that starting from a functional block diagram of an ICU mechanical ventilator and carrying a systematic analysis, the main function blocks were implemented in such a way that combinations of standard off-the-shelf pneumatic and electronic components could be used. No special parts need to be fabricated at all. These components are interconnected and then synchronized by ad hoc software to obtain a reliable working ICU ventilator that has an increased functionality of 8 modes of ventilation. Because of a wider variety of options, the use of extensively field-proven off-the-shelf commercial components assures better availability and lower costs when compared to proprietary parts common in conventional ICU mechanical ventilators, without sacrificing reliability.

Future work will be focused on consolidating and documenting the reliability of VEMERS, through controlled clinical tests. In addition, adaptations of VEMERS for use in anesthesiology, neonate, and transportation ventilators will be explored.

Finally, there is much to be done in generating procedures and devices to test mechanical ventilators and also in RT training. For this reason, this research team is working on devices to systematically test EUV and conventional ventilators in triggered mode and in pressure support for a variety of patient conditions.

## Figures and Tables

**Figure 1:** Evolution of the use of mechanical ventilators in Chile. Chilean Ministry of Health Official Report (in Spanish).

**Figure 2:** (a) VEMERS 1.0. (b) VEMERS 2.0. (c) Electronic circuits VEMERS 2.0. (d) Electropneumatic circuitry, valves, sensors, and parts. VEMERS 2.0.

**Figure 3:** Choked flow principle applied to mechanical ventilator inhalation phase.

**Figure 4:** Expiratory flow and pressure control.

**Figure 5:** Electropneumatic schematics of original VEMERS 1.0. Directional valves and manual flow control valves are used.

**Figure 6:** VEMERS 2.0. Upgraded mechanical ventilator schematics. Proportional valves have replaced directional valves and manual flow control valves in both the inhalation and expiratory phases of the cycle.

**Figure 7:** Patient curves in volume control mode (legends are in Spanish).

**Figure 8:** Patient curves in pressure control mode (legends in Spanish).

**Figure 9:** Patient curves in pressure support mode (legends are in Spanish).

**Figure 10:** Patient curves in CPAP mode of ventilation (legends in Spanish).

**Figure 11:** Typical patient curves in BiPAP mode of ventilation (legends in Spanish).

**Figure 12:** Typical patient curves in high-flow nasal cannula oxygenation mode of ventilation (legends in Spanish).

**Figure 13:** Pressure triggered assisted volume control mode of ventilation in VEMERS 2.0. The text is in Spanish to accommodate the RT native language.

**Figure 14:** Pressure triggered assisted pressure control mode of ventilation in VEMERS 2.0. The text is in Spanish to accommodate the RT native language.

**Figure 15:** Pressure support mode of ventilation in VEMERS 2.0. The text is in Spanish to accommodate the RT native language.

**Figure 16:** Different control range in two proportional valves. The range in SMC 2121-3 is much more desirable and allows more reliable and stable control of the mechanical ventilator.

**Table 1:** Working limits on VEMERS 2.0.

Limit	Units	Value
Maximum cycle volume	ml	800
Minimum cycle volume	ml	125
Failsafe relief pressure	cm H20	60
Maximum pressure in pressure control mode	cm H20	40
Minimum pressure in pressure control mode	cm H20 10	
Maximum peep	cm H20	25
Highest trigger pressure in assisted mode	cm H20	−3
Lowest trigger pressure in assisted mode	cm H20	−10
Maximum respiratory frequency	bpm	40
Minimum respiratory frequency	bpm	10
Maximum IE ratio		3
Minimum IE ratio		1
Maximum flow	lpm	60
Maximum time apnea in pressure support mode	sec	60
Minimum time apnea in pressure support mode	sec	5
Maximum flow O2 therapy	lpm	60
Minimum flow O2 therapy	lpm	10

**Table 2:** Ventilation modes in VEMERS 2.0. See [17] for a detailed description.

Mode number	Ventilation mode
1	Mandatory volume control
2	Assisted volume control triggered by pressure
3	Mandatory pressure control
4	Assisted pressure control triggered by pressure
5	Pressure support
6	CPAP
7	BiPAP
8	High oxygen flow therapy

**Table 3:** List of certifications for VEMERS project.

No.	Date	Type	Institution	Version	Comments
1	May 26, 2020	Technical validation	Certemed, University of Valparaiso	VEMERS 1.0	See [21]
2	May 28, 2020	Usability test	CMFCC	VEMERS 1.0	See [22]
3	June 9, 2020	Preclinic tests	Hospital Clinico UC Christus	VEMERS 1.0	See [23]
4	June 23, 2020	Technical validation	Certemed, University of Valparaiso	VEMERS 1.0	See [21]
5	August 3, 2020	Clinical tests	Hospital Clinico UC Christus	VEMERS 1.0,	Carried on 5 COVID-19 patients for 8 hours each. See [24–26]
6	March 21, 2021	Technical validation	Certemed, University of Valparaiso	VEMERS 2.0	Volume control modes. See [26]
7	April 14, 2021	Technical validation	Certemed, University of Valparaiso	VEMERS 2.0	Pressure control modes. See [26]

**Table 4:** Patient General Data in VEMERS UC Clinical tests.

Date	Testing hours	Volume (ml)	Frequency (bp)	IE ratio	PEEP (cm H_2_O)	Fio2	Patient age	Gender	Position
13/07/2020	13 : 20 to 21 : 20	280	32.0	2.0	8.0	45 a 60	62	male	Prono
17/07/2020	11 : 15 to 19 : 15	260	33.0	1.8	4.0	45 a70	70	Female	Prono
21/07/2020	10 : 00 to 18 : 00	360	20.0	2.1	10.0	35 a 40	72	Female	Supina
22/07/2020	9 : 00 to 17 : 00	340	28.0	1.9	6.0	45 a 60	59	Female	Supina
29/07/2020	13 : 20 to 20 : 00	275	29.7	1.9	7.9	50 a 55	72	Female	Supina

**Table 5:** VEMERS 2.0 distribution in the Chilean health system.

Regional health service	Quantity	Hospital	Date
Servicio de Salud Metropolitano Sur oriente	4	Sótero del Río (4)	April 1, 2021
Servicio de Salud del Maule	4	Curicó (2) and Linares (2)	April 12, 2021
Servicio de Salud de Coquimbo	4	La Serena (1), Coquimbo (1), Illapel (1), Ovalle (1)	April 19, 2021
Servicio de Salud de Ñuble	3	San Carlos (3)	May 7, 2021
Servicio de Salud Bío Bío, Concepción	2	Guillermo Grant Benavente (2)	June 1, 2021
Servicio de Salud Iquique	3	Iquique (3)	June 15, 2021

## Data Availability

All data are available upon request.

## Nomenclature

### Acronyms

BiPAP: Bilevel inhalation positive airway pressure
CPAP: Continuous positive airway pressure
CMFCC: Ad hoc committee to certify emergency mechanical ventilators in Chile
EUV: Emergency use ventilator
FiO2: Fraction of inhalation oxygen
HEPA: High-efficiency particulate air filter
I : E ratio: Inspiratory-expiratory time interval ratio
ICU: Intensive care unit
PEEP: Positive end-expiratory pressure
PIP: Peak inhalation pressure
RR: Respiration rate
RT: Respiratory therapist
SDV: Solenoid directional valve (ON-OFF)
SPV1: Solenoid proportional valve 1, controls the inspiratory flow
SPV2: Solenoid proportional valve 2, controls the expiratory flow
WHO: World Health Organization

### Variables

*A*_1_: Area of the aperture of valve SPV1 (mm^2^)
*A*_3_: Area of the aperture of valve SPV2 (mm^2^)
*C*_1_: Speed of gas mixture through valve SPV1
*C*_3_: Speed of gas mixture through valve SPV2
*c*_*p*_: Specific heat of air [Joule/(Kelvin · kg)]
*k*: Ratio of specific heats of air [ = 1.4]
*p*_0_: Pressure upstream of valve SPV1 [cm H20]
*p*_1_: Pressure at the aperture of valve SPV1 [cm H20]
*p*_2_: Patient lung pressure [cm H20]
*p*_*a*_: Absolute ambient pressure [cm H20]
*p* ^*∗*^: Critical pressure in choked flow [cm H20]
${\dot{Q}}_{1}$: Flow through SPV1 (lpm)
${\dot{Q}}_{3}$: Flow through SPV2 (lpm)
*R*: Air gas constant=287 [Joule/(Kelvin · kg)]
*T*_0_: Absolute temperature upstream of valve SPV1 (kelvin)
*ρ*_0_: Gas mixture density upstream of valve SPV1 [kg/*m*^3^].
